The article "Effects of microRNA-146a on the proliferation and apoptosis of human osteochondrocytes by targeting TRAF6 through the NF- κB signalling pathway" was retracted in 2021. Reason: citations of retracted work.

# Effects of microRNA-146a on the proliferation and apoptosis of human osteochondrocytes by targeting TRAF6 through the NF- κB signalling pathway

**DOI:** 10.1042/BSR20170180

**Published:** 2017-07-12

**Authors:** Camilla West, Michael F. McDermott

**Affiliations:** Leeds Institute of Rheumatic and Musculoskeletal Medicine (LIRMM), Wellcome Trust Brenner Building, St James University Hospital, University of Leeds, Leeds 32840, U.K.

**Keywords:** MicroRNA-146a, NF- κB, osteochondrocytes, Osteoarthritis

## Abstract

MicroRNAs are important cellular mediators of mRNA degradation and translation repression, which in turn can have an impact on various processes and, if their function is perturbed, can cause disease. Here, we summarize the recent manuscript by Zhong et al. [(2017) Biosci. Rep. **37**, BSR20160578], which explores microRNA-146a and how it may play an indirect yet vital role in the proliferation of osteoarthritis (OA) chondrocytes. The data presented by the authors could have important implications for future OA therapies.

Osteoarthritis (OA) is a chronic degenerative joint disease, characterized by synovial inflammation, deterioration of the articular cartilage and structural changes to the subchondral bone. Factors which increase the susceptibility to OA include ageing, obesity, genetics and joint injury. In 2005, it was estimated that 26 million people in the US alone had some form of OA [1] but despite this prevalence, treatment for OA remains unsatisfactory. There is a need for further research into understanding the pathogenesis and mechanisms of OA in order to identify new therapeutic targets. It has emerged in recent years that microRNAs (miRs) are involved in the onset and development of OA and can modulate various cellular processes, such as apoptosis, cell differentiation and proliferation, and matrix remodelling. The study by Zhong et al. [2] in this issue of *Bioscience Reports* examines the putative role of miR-146a in OA, via its regulation of TNF receptor-associated factor 6 (TRAF6) and the NF-κB signalling pathway, and also describes how the miR-146a–NF-κB–TRAF6 pathway may be a therapeutic target for OA.

miRs are known to have diverse roles in many cellular functions such as cell cycle control, apoptosis, development and metabolism. They are also known to be involved in immune regulation, and miR-146a has previously been reported to be up-regulated during toll-like receptor (TLR) signalling following lipopolysaccharide (LPS) stimulation [3], and to play a role in endotoxin tolerance [4]. With regards to OA, levels of miR-146a are known to be lower in the cartilage of patients with OA and to exercise control knee joint homoeostasis [5]. The use of histone deacetylase inhibitors, to increase miR-146a expression in OA synoviocytes, inhibited IL-1β-induced signalling and cytokine release, thereby lowering the level of inflammation [6]. The way in which miR-146a exerts these effects is by negative regulation of TRAF6 and IL-1 receptor-associated kinase 1 (IRAK1), both critical mediators of inflammation, via impairment of NF-κB activity [6,7]. This study by Zhong et al. further examined the role of miR-146a in the NF-κB–TRAF6 pathway, and its role in the proliferation and apoptosis of OA chondrocytes, in addition to highlighting further how this axis may provide a therapeutic target in OA [2].

The article "Effects of microRNA-146a on the proliferation and apoptosis of human osteochondrocytes by targeting TRAF6 through the NF- κB signalling pathway" was retracted in 2021. Reason: citations of retracted work.

Zhong et al. divided human OA and normal chondrocytes into seven groups: a normal group (normal chondrocytes), a blank group (OA chondrocytes without any transfection), a normal control (NC) group (OA chondrocytes transfected with nonsense sequences), an miR-146a mimics group (OA chondrocytes transiently transfected with miR-146a mimics plasmid), an miR-146a inhibitors group (OA chondrocytes transiently transfected with miR-146a inhibitors plasmid), an miR-146a inhibitor + si-TRAF6 group (OA chondrocytes transfected with miR-146a inhibitors plasmid and TRAF6 siRNA sequences) and an si-TRAF6 group (OA chondrocytes transfected with TRAF6 siRNA sequences) [2]. The authors first tested the possibility that TRAF6 is regulated post-transcriptionally by miR-146 in OA chondrocytes, by using reporter constructs which contained the luciferase gene fused to the 3′-UTRs from TRAF6, which contained the putative miR-146a target sites (originally reported in [3]). They observed a marked reduction in luciferase activity in chondrocytes expressing miR-146a and the TRAF6 construct, thereby suggesting that TRAF6 is subject to post-transcriptional repression by miR-146a. Following this, they also found that mRNA expression of TRAF6 and NF-κB was decreased in the miR-146a mimics group but was increased in the miR-146a inhibitors group. This regulation of TRAF6 and NF-κB by miR-146a was further validated by Western blotting, where cells overexpressing miR-146a displayed a decrease in both TRAF6 and NF-κB expression at the protein level. Their next steps were to look at the functional relevance of this modulation of TRAF6 and NF-κB by miR-146a, and the authors chose to look at differences in cell proliferation and apoptosis among the seven groups of chondrocytes. They found that miR-146a enhances proliferation and that this may be via suppression of TRAF6. Furthermore, they provide evidence for a role for miR-146a in apoptosis, as chondrocytes overexpressing miR-146a had reduced levels of cellular apoptosis. This study is not the first to look at miR-146a in relation to apoptosis and proliferation; it is known that this non-coding RNA has an anti-inflammatory role in dendritic cells and the miR-146a–TRAF6–NF-κB pathway has been recently shown to be responsible for dendritic cell apoptosis [8]. This miRNA has also been studied in the context of cancer and, depending on cell type, can either up-regulate or down-regulate apoptosis and proliferation. For example, miR-146a was shown to be associated with suppression of breast cancer metastases via the down-regulation of epidermal growth factor receptor (EGFR) [9]. Thus, it will be pertinent in future studies of miR-146a in OA to examine the EGFR and other pathways involved in cellular growth and proliferation.

The article "Effects of microRNA-146a on the proliferation and apoptosis of human osteochondrocytes by targeting TRAF6 through the NF- κB signalling pathway" was retracted in 2021. Reason: citations of retracted work.

Overall, this study provides compelling data to support a novel role of miR-146a in targeting TRAF6, via the NF-κB pathway, in the context of OA chondrocyte proliferation and apoptosis. miRNA-146a inhibited protein expression of TRAF6 and NF-κB in OA chondrocytes and, importantly, this negative regulation of TRAF6 led to increased proliferation of OA chondrocytes. Heightened proliferation of OA chondrocytes has been purported to have a positive impact on joint repair, thus this is an exciting development in understanding this mechanism [10]. If progressed further, this finding could have significant therapeutic implications for OA. miRNAs can be specifically inhibited by chemically modified antisense oligonucleotides, and this gives a promising outlook for miRNA-based therapies for many diseases, including cancer, autoimmune and cardiovascular diseases. In recent years, specific antagonists for miRNAs (antagomirs) have been developed including, for example, anti-miR-155 for rheumatoid arthritis [11]. miRNA replacement therapy is another potential strategy, where exogenous miRNAs are administered to substitute for endogenous miRNAs [12]. The potential of these therapies will remain unproven until developments in the design of miRNA small molecule inhibitors and improved methods for their *in vivo* delivery are made. Nevertheless, this could be an exciting alternative to other therapeutic options, such as gene therapy, and will have broad implications for many human diseases, including OA.

This study makes a case for the therapeutic potential of miR-146a in OA, by promoting the proliferation of OA chondrocytes, with inhibiting apoptosis of these cells, thereby protecting articular cartilage in OA. This study will stimulate further research into these other miR-146a targets, by evaluating how these are regulated and altered in OA, and is likely to contribute to a much-improved understanding of this debilitating condition.

The article "Effects of microRNA-146a on the proliferation and apoptosis of human osteochondrocytes by targeting TRAF6 through the NF- κB signalling pathway" was retracted in 2021. Reason: citations of retracted work.

## Abbreviations

EGFR: epidermal growth factor receptor
IL-1beta: interleukin-1 beta
IRAK1: IL-1 receptor-associated kinase 1
LPS: lipopolysaccharide
OA: osteoarthritis
TLR: toll-like receptor
TNF: tumor necrosis factor
